The article "Flexible Ureteroscopy and Nephroscopy for Stone Removal in Patients with Multiple Renal Calculi" was retracted in 2023. Reasons: signs of a paper mill; suspected computer-generated content; unreliable results or conclusions; lack of ethics approval or compliance.

# Flexible Ureteroscopy and Nephroscopy for Stone Removal in Patients with Multiple Renal Calculi

**DOI:** 10.1155/2022/2078979

**Published:** 2022-07-09

**Authors:** Bin Zhu, Suibing Zhang

**Affiliations:** Pingshan District People's Hospital of Shenzhen, Pingshan General Hospital of Southern Medical University, Shenzhen, Guangdong 518118, China

## Abstract

**Objective:**

Renal calculi are a common type of urological calculi and are associated with morbidity. This study was aimed at exploring the effect of flexible ureteroscopy and nephroscopy on stone removal in patients with multiple renal calculi.

**Method:**

This randomized controlled trial included a total of 78 cases with multiple renal calculi in our hospital. The patients were randomly divided into the study and control groups and treated with flexible ureteroscopy and percutaneous nephrolithotomy with pneumatic ballistics, respectively. The surgery condition, levels of prostaglandin F2*α* (PGF2*α*), prostaglandin E2 (PGE2), keratocyte growth factor (KGF), renal function indices, and the incidence of complications were analyzed before and after surgery in the two groups.

**Result:**

The operation time, the postoperative analgesia pump application time, one-time stone removal rate, the intraoperative blood loss, and hospital stay of the study group were significantly lower than those of the control group. Postsurgery, the levels of PGE2, PGF2*α,* and KGF in the study group were significantly lower than those in the control group. The serum levels of SCR, BUN, and NGAL in the study group were significantly lower than those in the control group. In addition, the incidence complications in the study group were significantly lower.

**Conclusion:**

Flexible ureteroscopy and laser lithotripsy under nephroscopy were equally effective against multiple renal calculi. Flexible ureteroscopy reduced surgical trauma without affecting renal function and had a low incidence of complications.

## 1. Introduction

Due to changes in the dietary habits of the modern population, the incidence of urinary tract stones is increasing year by year. Previous studies have shown that kidney stones are a common type of urinary tract stones. Multiple kidney stones are usually accompanied by varying degrees of severe pain in the upper abdomen or waist that continues to spread. If patients do not receive timely and effective intervention, irreversible damage to the kidneys will occur [1–3]. Therefore, early intervention is of great significance for patients with multiple nephrolithiasis.

Although surgical intervention is the main treatment method for multiple kidney stones, traditional surgical methods have the disadvantages of high infection risk, low stone clearance rate, and high recurrence rate, which limit their clinical application [4, 5]. In recent years, with the improvement and popularization of minimally invasive techniques, flexible ureteroscopy can reduce surgical trauma and complications and has been widely used in the treatment of multiple kidney stones [6, 7].

The article "Flexible Ureteroscopy and Nephroscopy for Stone Removal in Patients with Multiple Renal Calculi" was retracted in 2023. Reasons: signs of a paper mill; suspected computer-generated content; unreliable results or conclusions; lack of ethics approval or compliance.

In this study, we aimed to explore the effect of flexible ureteroscopy and nephroscopy on stone removal in patients with multiple renal calculi.

## 2. Material and Methods

### 2.1. Patient Selection Criteria

The inclusion criteria for this study were as follows: (1) the patient was diagnosed with multiple nephrolithiasis by urology CT, venography, and B-ultrasound; (2) the patient was aware of this study and signed the informed consent; (3) age ≤ 70 years; (4) first received surgical treatment patients; and (5) patients with surgical indications. The exclusion criteria for this study were (1) patients with urinary tract infection; (2) patients with previous renal insufficiency, nephritis, and other renal diseases; (3) patients with pulmonary and cardiac insufficiency; (4) patients with complications of urinary tract tumors; and (5) patients with contraindications.

### 2.2. Method

Patients in the study group were treated with flexible ureteroscopes and flexible ureteroscope negative pressure sheaths (Kangyi Company, China). The patient received general anesthesia with endotracheal intubation and took the lithotomy position. The flexible ureteroscope negative pressure cannula was indwelled retrogradely, and the flexible ureteroscope negative pressure cannula was placed into the bladder for exploration. The ipsilateral ureteral opening was defined along the interureteric ridge, and the lens was introduced into the renal pelvis through a guide wire. Determine the location of the stone, and insert the holmium laser fiber through the ureteroscope surgical channel. Central lithotripsy and peripheral lithotripsy were used to crush stones, and ureteral stents were retrogradely placed in the paralithic space with the largest stone fragment < 3 mm. After that, the gravel was taken out, the holmium laser fiber was taken out, the flexible ureteroscope were taken out, and the double J tube was inserted. In the control group, pneumatic ballistic percutaneous nephrolithotomy was used. The patient received general anesthesia and was placed in the lithotomy position. Cystoscope is retrogradely cannulated from the affected ureter and the catheter tip is secured. Move the patient to the prone position with the affected side elevated 20°. The selected puncture site was the intersection of the subscapular angle line, the posterior axillary line, and the 11th to 12th intercostal regions. An appropriate amount of normal saline was injected into the ureteral catheter to establish an artificial hydronephrosis channel. The puncture was performed under ultrasound guidance, and a percutaneous nephroscope was inserted under a low-pressure perfusion environment to establish a percutaneous nephroscope. Use a pneumatic lithotripsy to locate and remove stones. Large stones were taken out with forceps, and small stones were rinsed with normal saline. Postoperatively, residual stones were checked and the fistula was fixed. Antibiotics were routinely used postoperatively. The indwelling catheter was removed 3 to 5 days after the operation, and the stones were checked regularly after the operation.

The article "Flexible Ureteroscopy and Nephroscopy for Stone Removal in Patients with Multiple Renal Calculi" was retracted in 2023. Reasons: signs of a paper mill; suspected computer-generated content; unreliable results or conclusions; lack of ethics approval or compliance.

### 2.3. Outcome Parameters

(1) The surgical conditions, including operative time, postoperative analgesia pump application time, one-time stone clearance rate, intraoperative blood loss, and length of hospital stay, were evaluated in both groups. (2) The levels of prostaglandin F2*α* (PGF2*α*), prostaglandin E2 (PGE2), and keratin growth factor (KGF) in the two groups before and after the operation were measured. Peripheral blood (3 mL) was extracted and centrifuged (3500 r/min, 15 min) to obtain the supernatant. An enzyme-linked immunosorbent assay (ELISA) was performed using Bio-Rad 550 enzyme plate analyzer and kit. (3) Renal function before and after the operation in the two groups was evaluated by measuring (blood urea nitrogen (BUN), serum creatinine (SCR), and gelatinase-associated lipid carrier protein (NGAL)). (4) Incidence of complications in the two groups was recorded.

### 2.4. Statistical Analysis

The data was analyzed by SPSS Statistics 22.0 (IBM Corp., Armonk, N.Y., USA). Measurement data was presented as mean ± standard deviation. The differences were tested by *t-*test. *P* < 0.05 was considered statistically significant.

## 3. Results

### 3.1. Baseline Data

In this study, 78 patients with multiple renal calculi admitted to our hospital from January 2019 to March 2021 were selected and randomly divided into the study group (*n* = 39) and the control group (*n* = 39) according to the simple random number table method. The study group consisted of 26 males and 13 females, with an average age of 53.45 ± 6.02 years, ranging from 38 to 69 years old. The diameter of the stones was 1.2 to 2.7 cm, with an average of 1.95 ± 0.41 cm. The number of stones ranged from 2 to 11, with an average of 6.45 ± 3.01. The course of disease was 1.5 to 6.6 years, with an average of 4.05 ± 1.08 years. Body mass index (BMI) was 18.2 − 28.9 kg/m^2^, with an average of 23.55 ± 2.96 kg/m^2^. The control group consisted of 28 men and 11 women. The average age was 55.02 ± 5.67 years, ranging from 36 to 70 years old. The diameters of the stones ranged from 1.1 to 2.9 cm, with an average of 2.02 ± 0.39 cm. The number of calculi ranged from 2 to 13, with an average of 7.04 ± 2.98. The course of disease was 1.3 to 7.5 years, with an average of 3.98 ± 1.11 years. BMI ranged from 17.8 to 29.7 kg/m^2^ with a mean of 24.14 ± 3.03 kg/m^2^. There were no significant differences in clinical characteristics such as gender, age, stone diameter, course of disease, number of stones, and BMI between the two groups (*P* > 0.05).

The article "Flexible Ureteroscopy and Nephroscopy for Stone Removal in Patients with Multiple Renal Calculi" was retracted in 2023. Reasons: signs of a paper mill; suspected computer-generated content; unreliable results or conclusions; lack of ethics approval or compliance.

### 3.2. Comparison of Surgical Conditions between the Two Groups

As shown in Table 1, the operation time, the postoperative analgesia pump application time, one-time stone removal rate, the intraoperative blood loss, and hospital stay of the study group were significantly lower than those of the control group (*P* < 0.05).

### 3.3. Comparison of PGF2*α*, PGE2, and KGF before and after Surgery between the Two Groups

The serum levels of PGE2 (138.56 ± 20.12 pg/mL), PGF2*α* (82.56 ± 10.27 ng/mL), and KGF (0.58 ± 0.11 ng/mL) in the study group were comparable to those in the control group (141.97 ± 22.68 pg/mL, 84.05 ± 11.12 ng/mL, and 0.60 ± 0.09 ng/mL). The serum levels of PGF2*α*, PGE2, and KGF in both groups after surgery were higher than those before operation (*P* < 0.05). However, as shown in Table 2, postsurgery, the levels of PGE2 (169.45 ± 21.15 pg/mL), PGF2*α* (103.34 ± 17.13 ng/mL), and KGF (0.79 ± 0.14 ng/mL) in the study group were significantly lower (*P* < 0.05) than those in the control group (212.30 ± 24.68 pg/mL, 136.71 ± 21.40 ng/mL, and 1.02 ± 0.16 ng/mL).

### 3.4. Comparison of Renal Function Indices between Groups

As shown in Table 3, preoperative serum levels of SCR (75.58 ± 9.67 *μ*mol/L), BUN (6.41 ± 1.40 mmol/L), and NGAL (3.89 ± 0.77 *μ*g/L) in the study group were comparable to those in the control group (SCR: 73.71 ± 10.32 *μ*mol/L, 6.55 ± 1.38 mmol/L, and 3.93 ± 0.80 *μ*g/L, respectively). The serum levels of Scr, BUN, and NGAL in the two groups after surgery were higher than those before surgery (*P* < 0.05). Postsurgical serum levels of SCR (86.11 ± 9.04 *μ*mol/L), BUN (7.40 ± 1.12 mmol/L), and NGAL (6.11 ± 0.93 *μ*g/L) in the study group were significantly lower (*P* < 0.05) than those in the control group (SCR: 99.37 ± 8.91 *μ*mol/L, 8.96 ± 1.23 mmol/L, and 8.79 ± 1.02 *μ*g/L).

### 3.5. Comparison of the Incidence of Complications between the Two Groups

The incidence of complications in the study group was significantly lower than in the control group (5.13% vs. 23.08%, *P* < 0.05; Table 4).

The article "Flexible Ureteroscopy and Nephroscopy for Stone Removal in Patients with Multiple Renal Calculi" was retracted in 2023. Reasons: signs of a paper mill; suspected computer-generated content; unreliable results or conclusions; lack of ethics approval or compliance.

## 4. Discussion

Multiple renal calculi are associated with relatively high morbidity. The primary treatment still remains surgery, with open surgery having significant effectiveness. However, only multiple incisions in the kidney can ensure stone removal, leading to greater trauma and more complications, which is not conducive to postoperative functional rehabilitation [8, 9]. Extracorporeal shock wave lithotripsy plays a vital role in treating multiple renal calculi, but its therapeutic effect is affected by the stone size and location [10]. Therefore, a safe and effective treatment strategy for multiple renal calculi is still missing.

With recent technological improvements, although flexible ureteroscopy has gradually become a common treatment for multiple renal calculi, the value of flexible ureteroscopy in multiple renal calculi lacks sufficient evidence-based research [11]. In order to serve as a reference for the clinical selection of reasonable surgical methods, our study covered several aspects. In the present study, flexible ureteroscopy and percutaneous nephrolithotomy were used to treat patients with multiple renal calculi. Our results showed that although the two methods had a similar removal rate effect, flexible ureteroscopy had a significant advantage in reducing surgical trauma by reducing the damage to renal function and shortening postoperative rehabilitation [12–14]. However, the flexible ureteroscope can retrograde into the ureter, renal pelvis, and renal calyces through the natural body cavities, more consistent with the physiological characteristics of the human body, thus avoiding damage to body organs and tissues [12, 15]. Moreover, when the ureter is severely obstructed or distorted, a flexible ureteroscope can be adopted for treatment, convenient to avoid blind operation and damage to the kidney and other functions. Furthermore, a flexible ureteroscope has a higher definition and flexibility and can help perform the operation with minimal invasiveness through the human natural cavity, thus minimizing the impact of the invasive operation on renal parenchymal injury and renal function [16, 17]. Meanwhile, although ureteroscopy has the advantage of being less invasive, it can also damage kidney function due to its thinness because when the fluid pressure in the renal pelvis is high, it cannot be restored in time. As a result, the perfusion pressure in the renal pelvis increases, leading to a reflux phenomenon, which aggravates glomerular damage, causing renal injury [18, 19].

In addition, although flexible ureteroscopy is less traumatic, it is still an aggressive treatment, which can cause elicit different degrees of inflammatory stress responses. Furthermore, inflammatory stress response may cause postoperative adhesion to endothelial function, renal function, and others, leading to damage and circulatory dysfunction. This can lead to an increased PGF2*α*, PGE2, and KGF pain media production, which cause vasoconstriction and can cause an inflammatory reaction, thus increasing blood vessel permeability. It can also activate slow excitation peptide, which causes tissue edema and pain, and its serum level is closely related to the degree of pain. This study showed that PGF2*α*, PGE2, and KGF serum levels in the study group were significantly lower than those in the control group (*P* < 0.05), further demonstrating the higher application value of flexible ureteroscopy in patients with multiple renal calculi. Further, we found a lower incidence of complications in the study group than in the control group, further confirming the safety of flexible ureteroscopy in treating multiple renal calculi.

The article "Flexible Ureteroscopy and Nephroscopy for Stone Removal in Patients with Multiple Renal Calculi" was retracted in 2023. Reasons: signs of a paper mill; suspected computer-generated content; unreliable results or conclusions; lack of ethics approval or compliance.

In conclusion, flexible ureteroscopy and laser lithotripsy under nephroscopy were similarly efficacious in patients with multiple renal calculi. However, flexible ureteroscopy reduced surgical trauma, inhibited the pain and stress caused by surgical trauma, and had smaller effects on renal function and incidence of complications was low.

## Figures and Tables

**Table 1:** Comparison of surgical conditions between the two groups.

Groups	Cases	The operative time (min)	The postoperative analgesia pump application time (d)	One-time stone removal rate (%)	The intraoperative blood loss (mL)	The hospital stay (d)
The study group	39	51.63 ± 10.69	2.06 ± 0.59	36 (92.31)	14.09 ± 3.68	3.41 ± 0.83
The control group	39	64.34 ± 12.56	2.81 ± 0.64	34 (87.18)	21.68 ± 5.11	5.56 ± 0.97
*t/χ* ^2^ value		4.812	5.381	0.557	7.527	10.517
*P* value		0.231	0.407	0.455	0.032	0.014

**Table 2:** Comparison of PGF2*α*, PGE2, and KGF before and after surgery between groups.

Time	Groups	Cases	PGE2 (pg/mL)	PGF2*α* (ng/mL)	KGF (ng/mL)
Before the operation	The study group	39	138.56 ± 20.12	82.56 ± 10.27	0.58 ± 0.11
	The control group	39	141.97 ± 22.68	84.05 ± 11.12	0.60 ± 0.09
	*t* value		0.702	0.615	0.879
	*P* value		0.585	0.541	0.682
After the operation	The study group	39	169.45 ± 21.15	103.34 ± 17.13	0.79 ± 0.14
	The control group	39	212.30 ± 24.68	136.71 ± 21.40	1.02 ± 0.16
	*t* value		8.233	7.602	6.756
	*P* value		0.015	0.019	0.012

PGF2*α*: prostaglandin F2*α*; PGE2: prostaglandin E2; KGF: keratin growth factor.

**Table 3:** Comparison of renal function indices between groups.

Time	Groups	Cases	BUN (mmol/L)	Scr (*μ*mol/L)	NGAL (*μ*g/L)
Before the operation	The study group	39	6.41 ± 1.40	75.58 ± 9.67	3.89 ± 0.77
	The control group	39	6.55 ± 1.38	73.71 ± 10.32	3.93 ± 0.80
	*t* value		0.445	0.826	0.225
	*P* value		0.658	0.612	0.823
After the operation	The study group	39	7.40 ± 1.12	86.11 ± 9.04	6.11 ± 0.93
	The control group	39	8.96 ± 1.23	99.37 ± 8.91	8.79 ± 1.02
	*t* value		5.856	6.524	12.125
	*P* value		0.321	0.439	0.387

BUN: blood urea nitrogen; NGAL: gelatinase-associated lipid carrier protein; SCR: serum creatinine.

The article "Flexible Ureteroscopy and Nephroscopy for Stone Removal in Patients with Multiple Renal Calculi" was retracted in 2023. Reasons: signs of a paper mill; suspected computer-generated content; unreliable results or conclusions; lack of ethics approval or compliance.

**Table 4:** Comparison of the incidence of complications between groups *n* (%).

Groups	Cases	Fever	Ureteral mucosa injury	Urinary tract infection	Hematuresis	The total incidence
The study group	39	1 (2.56)	0 (0.00)	1 (2.56)	0 (0.00)	2 (5.13)
The control group	39	2 (5.13)	2 (5.13)	3 (7.69)	2 (5.13)	9 (23.08)
*χ* ^2^ value						5.186
*P* value						0.023

## Data Availability

All data was within the manuscript.
